# Diagnostic and Prognostic Nomograms for Lung Metastasis in Triple-Negative Breast Cancer

**DOI:** 10.1155/2022/1750834

**Published:** 2022-08-11

**Authors:** Jianguo Wang, Hongjun Zhao, Lifen Ye, Jingyong Li, Huaixiao Zhang, Chao Zhang, Qishuo Rao, Yurong Cai, Yiping Xu, Youyuan Deng

**Affiliations:** Department of General Surgery, Xiangtan Central Hospital, Xiangtan, China

## Abstract

**Background:**

The lungs are one of the common sites of metastasis of triple-negative breast cancer (TNBC). Patients with lung metastases (LM) have a shorter duration of survival. This study is aimed at determining the prognostic factors of patients with TNBC with LM and constructing two nomograms to assess the risk of LM and the prognosis of patients with TNBC with LM.

**Methods:**

Clinicopathological and follow-up data of patients with TNBC between 2010 and 2015 were retrieved from the Surveillance, Epidemiology, and End Results (SEER) database. Univariate and multivariate Cox regression analyses were used to screen for independent predictors of LM in patients with TNBC and identify the independent prognostic factors of patients with TNBC with LM. The two nomograms were appraised using calibration curves, receiver operating characteristic (ROC) curves, and decision curve analysis (DCA).

**Results:**

A total of 27,048 patients with TNBC were included in this study. Age, tumour size, T stage, and N stage were identified as independent risk factors for LM in patients with TNBC. Histological type, marital status, prior surgery, chemotherapy, bone metastases, brain metastases, and LM were confirmed as independent prognostic factors for patients with TNBC with LM. The area under the ROC curve (AUC) of the diagnostic nomogram was 0.838 (95% confidence interval 0.817-0.860) in the training cohort and 0.894 (95% confidence interval 0.875-0.917) in the verification cohort. The AUC values of the 6-, 12-, and 18-month prognostic nomograms in the training cohort were 0.809 (95% confidence interval 0.771-0.868), 0.779 (95% confidence interval 0.737-0.834), and 0.735 (95% confidence interval 0.699-0.811), respectively, and the corresponding AUC values in the validation cohort were 0.735(95% confidence interval 0.642-0.820), 0.672 (95% confidence interval 0.575-0.758), and 0.705 (95% confidence interval 0.598-0.782), respectively. According to the calibration curves and data analysis, both nomograms exhibited good performance.

**Conclusion:**

We successfully constructed and verified two valuable nomograms for predicting the incidence of LM and prognosis of patients TNBC with LM.

## 1. Introduction

Breast cancer is the most common malignant tumour in women, and breast cancer-specific deaths accounted for approximately 15% of cancer-related deaths in women in 2018 [1]. Triple-negative breast cancer (TNBC) accounts for approximately 10–20% of all breast cancer cases [2, 3]. Chemotherapy is the mainstay of treatment for TNBC because of the lack of expression of oestrogen receptor (ER), progesterone receptor (PR), and human epidermal growth factor receptor 2 (HER2) in patients [4]. Patients with TNBC have a worse prognosis than those with other types of breast cancer and have a mortality rate of 40% within the first 5 years of diagnosis [5].

Moreover, approximately 50% of patients with TNBC develop distant metastasis [6]. The mortality rate of patients with distant metastases is higher than that of patients with carcinoma in situ [7]. The lungs are one of the most common sites of distant metastasis, accounting for 40% of the cases of metastasis. The median survival time of patients with metastatic TNBC is 1–1.5 years [8]. Therefore, determining a new method to predict the risk of lung metastasis (LM) and the prognosis of patients with TNBC is extremely important. ENY2, KCNK9, TNFRSF11B, KXNMB2, race, and marital status have been identified as risk factors and prognostic variables of LM [9, 10]. To the best of our knowledge, no in-depth studies performed thus far have used predictive models to determine the incidence and prognosis of TNBC with LM; therefore, risk factors cannot be combined to effectively assess individual outcomes, and implementation of precision medicine is thus hampered.

A nomogram is a convenient tool that can accurately predict individual outcomes and exhibit good accuracy in assessing the prognosis of various cancers [11]. In this study, we aimed to construct two nomograms to predict the risk of LM in patients with TNBC and the prognosis of these patients based on the data from the Surveillance, Epidemiology, and End Results (SEER) database.

## 2. Methods

### 2.1. Study Population Selection

The SEER∗Stat software (version 8.3.6) was used to download patient data from the SEER database. Patients diagnosed with TNBC from 2010 to 2015 were included in this study. The exclusion criteria were as follows: (1) patients in whom TNBC was not the primary tumour; (2) death of patients with an unknown cause; and (3) patients with unknown information, including age, tumour size, race, grade, histological type, T stage, N stage, LM, insurance status, and marital status. Eventually, 27,048 patients in the cohort were enrolled to examine the risk factors of TNBC with LM and establish a predictive nomogram. Subsequently, patients with TNBC with LM who survived ≥1 month; underwent surgery, radiotherapy, and chemotherapy; and had specific metastasis data, including bone, brain, and liver metastases, were included to form a new cohort to identify the prognostic factors of TNBC with LM and establish a prognostic nomogram. Eventually, we included 480 patients to investigate the prognostic factors of TNBC with LM; these patients were randomly divided into the training and validation cohort in a ratio of 7 : 3 (caret package (version: 6.0.88) of the R studio). The training cohort was used to develop a nomogram, which was externally verified in the verification cohort.

### 2.2. Data Collection

We used demographic variables, including age, race, insurance status, marital status, tumour characteristics, tumour size, grade, histological type, T stage, and N stage, to identify the risk factors of TNBC with LM. Additionally, we used data pertaining to metastasis to the bone, brain, and liver and treatment modalities, including surgery, chemotherapy, and radiotherapy, to determine the prognostic factors associated with TNBC with LM.

### 2.3. Statistical Analysis

All statistical analyses were performed using SPSS 25.0 and R software (version 3.6.1). A *P* value < 0.05 (bilateral) was considered statistically significant. Univariate logistic analysis and multivariate binary logistic regression analysis were performed to determine the independent risk factors of TNBC with LM. Univariate and multivariate Cox regression analyses were performed to identify the independent prognostic factors.

The receiver operating characteristic (ROC) curve and time-dependent ROC curve of the predicted nomogram were generated. The area under the ROC curve (AUC) signified the distinctiveness of the nomogram and was further compared with the AUC of all independent prognostic factors. In addition, calibration curves were established to compare the consistency between the actual results and those predicted by the line graph. The range of threshold probability and the size of benefits were determined using decision curve analysis (DCA). In addition, patients were divided into the high- and low-risk groups based on the median risk score. Kaplan–Meier (KM) curves were generated, and the logarithmic rank test was performed.

## 3. Results

### 3.1. Baseline Characteristics of Patients

The baseline characteristics of 27,048 patients with TNBC are shown in Table 1. The tumour size of most patients with TNBC was <5 cm, and of all patients, 19,402 (71.7%), were Caucasian. Most patients (80.3%) had stage III disease.

### 3.2. Risk Factors of TNBC with LM

To determine the LM-related variables of TNBC, we used single-factor logistic analysis to screen for risk factors and found that the age, tumour size, histological type, T stage, N stage, insurance status, and marital status of patients with TNBC were related to LM (Table 2). Furthermore, multivariate logistic analysis showed that age, tumour size, T stage, and N stage were independent predictors of LM in patients with TNBC (Table 2).

### 3.3. Construction and Validation of a Diagnostic Nomogram for TNBC with LM

The diagnostic nomogram of LM for patients with TNBC was constructed by including the corresponding independent risk factors (Figure 1). The AUC values of the training and verification cohort were 0.838 (95% confidence interval 0.817-0.860) and 0.894 (95% confidence interval 0.875-0.917), respectively (Figures 2(a) and 2(d)). Additionally, we generated ROC curves for each independent predictor (Figure 3) and found that the AUC of the nomogram was higher than that of all individual predictors. In addition, the calibration curve showed consistent results in the training and validation cohorts (Figures 2(b) and 2(e)). The DCA curve showed that the nomogram had high accuracy for the diagnosis of TNBC with LM (Figures 2(c) and 2(f)).

### 3.4. Prognostic Factors of TNBC with LM

To determine the prognostic factors, we examined the data from 480 patients with TNBC with LM (Table 3). Of these patients, 324 (67.5%) were Caucasian, 120 (25.0%) were Black, and 36 (7.5%) belonged to other races. Most patients received radiotherapy. Univariate and multivariate Cox proportional hazards regression were used to identify histological type, prior surgery, chemotherapy, bone metastasis, brain metastasis, liver metastasis, and marital status as independent prognostic factors of TNBC with LM (Table 4).

### 3.5. Construction and Validation of a Prognostic Nomogram for TNBC with LM

By integrating the identified independent prognostic factors, a prognostic nomogram was established for TNBC with LM (Figure 4). The AUC values for predicting prognosis at 6, 12, and 18 months were 0.809 (95% confidence interval 0.771-0.868), 0.779 (95% confidence interval 0.737-0.834), and 0.735 (95% confidence interval 0.699-0.811), respectively, in the training cohort and 0.735 (95% confidence interval 0.642-0.820), 0.672 (95% confidence interval 0.575-0.758), and 0.705 (95% confidence interval 0.598-0.782), respectively, in the verification cohort (Figures 5(a) and 5(c)). In addition, in the training and validation cohorts, the probability calibration curves for 6, 12, and 18 months showed good agreement (Figures 6(a) and 6(c)). The DCA curve showed that the predictive performance of the nomogram was relatively accurate (Figures 6(b) and 6(d)).

### 3.6. Comparison of Discrimination between Prognostic Nomogram and Independent Prognostic Factors

To assess the advantages of the prognostic nomogram, we generated ROC curves inclusive of independent prognostic factors and found that the AUC value of part prognostic factor was >0.650, which signified that part individual factors can be used as reliable prognostic factors. However, the AUCs of all prognostic factors were lower than those of the prognostic nomogram (Figure 7). Overall, we confirmed that the function of a rosette combining different information from individual patients is superior to the predictive power of evaluating individual risk factors.

### 3.7. Role of Prognostic Nomograms in Risk Stratification of Patients with TNBC with LM

The overall prognostic score of all patients TNBC with LM was calculated based on the nomogram. The KM curve showed that patients in the low-risk group survived longer than those in the high-risk group (Figures 5(b) and 5(d)). The threshold values identified in the training cohort were used for the validation cohort. The prognosis in both risk groups was significantly different (*P* < 0.0001). Overall, our system of risk stratification worked very well.

## 4. Discussion

TNBC is an aggressive tumour, which is prone to distant metastasis [12]. The lungs are a common site for distant metastasis. In this study, we constructed a diagnostic and a prognostic nomogram to predict LM in patients with TNBC. The risk of LM can be easily identified using these nomograms. The prognostic nomogram was used to assess the prognosis of TNBC patients with LM and provide guidance for further clinical management. The two nomograms accurately assessed the risk of LM and predicted survival and may help clinicians in decision-making and disease monitoring.

Although the prognosis of patients with TNBC with LM is extremely poor, early detection of LM is essential for patients to receive appropriate treatment [13]. Therefore, identifying risk factors of TNBC with LM is very important to guide clinical treatment. Several biomarkers and prognostic factors have been identified, including linc-ZNF469-3, miR-629-3p, age, T stage, and N stage [14–17]. However, to the best of our knowledge, no risk-prediction nomograms have been constructed to date; therefore, individual risk of LM cannot be quantified. Our results showed that age, tumour size, T stage, and N stage are independent predictors of TNBC with LM, which is consistent with the results of previous studies.

In addition, our results showed that patients with invasive ductal carcinoma (IDC), who were married, with no brain metastases, no liver metastases, and no bone metastases had a better prognosis after undergoing surgery and chemotherapy. Based on seven independent prognostic factors, a prognostic nomogram was constructed, which can be used as an effective tool to identify high-risk patients. IDC is the most common histological type of patients with TNBC [18]. Zhao et al. [19] and Li et al. [20] reported that the survival rate of patients with IDC is higher than that of patients with other histological types. These findings are consistent with those reported in our study. Patients who were married had a better prognosis. Previous studies have shown that the risk of cancer metastasis and cancer-related deaths is lower in married patients than in unmarried patients [21]. This relationship may be attributed to the important role of marital status in regulating the functions of the endocrine and immune systems [22]. Moreover, TNBC has a high recurrence rate [12]. We found that patients with distant metastases had a lower survival rate, which was consistent with the results of a study by Wang et al. [23]. In addition, different sites of metastasis affect the survival of patients with TNBC. Studies have reported that the prognosis of patients with visceral metastasis is worse than that of patients with bone metastasis [24]. Typically, the treatment of patients with advanced disease should focus on improving the survival rate of these patients. Chemotherapy and surgery are both favourable prognostic factors for patients with TNBC with LM. In addition, previous studies have shown that chemotherapy and surgery can significantly improve the prognosis of patients with LM [25]. Currently, chemotherapy remains the standard treatment for patients with TNBC [26]. The NCCN guidelines recommend a combination treatment plan based on taxanes, anthracycline, cyclophosphamide, cisplatin, and fluorouracil [6]. Previous studies have shown that despite metastasis to distant organs, patients can benefit from surgery [27, 28]. Our prognostic nomogram showed that surgery and chemotherapy were beneficial for the survival of patients with TNBC with LM. Therefore, identification of independent prognostic factors may help to identify high-risk patients and establish a specific monitoring plan.

However, our study has several limitations. The SEER database contains data regarding the first diagnosis of the disease; therefore, LM that occurs in advanced stages cannot be recorded. Furthermore, this is a retrospective study with large sample size; therefore, selection bias is inevitable. The prognostic nomogram was constructed and verified at a single institution, which may affect its clinical applicability to a certain extent. Therefore, further calibration of the nomogram is required in future studies.

## 5. Conclusion

Age, tumour size, T stage, and N stage are the risk factors of TNBC with LM. Histological type, marital status, brain metastasis, liver metastasis, bone metastasis, surgery, and chemotherapy are independent prognostic factors. The results of this study are very useful for determining individualised treatment and ensuring appropriate management of patients with TNBC with LM.

## Figures and Tables

**Figure 1:** Diagnostic nomogram of LM for patients with TNBC. LM: lung metastasis; TNBC: triple-negative breast cancer.

**Figure 2:** ROC curves (a), calibration curve (b), and DCA curve (c) of the diagnostic nomogram for patients with TNBC with LM in the training cohort. ROC curves (d), calibration curve (e), and DCA curve (f) of the diagnostic nomogram for patients with TNBC with LM in the validation cohort. ROC: receiver operating characteristic; DCA: decision curve analysis; LM: lung metastasis; TNBC: triple-negative breast cancer.

**Figure 3:** Independent predictor of ROC curves in the training cohort (a) and validation cohort (b). ROC: receiver operating characteristic.

**Figure 4:** Prognostic nomogram for patients with TNBC with LM. LM: lung metastasis; TNBC: triple-negative breast cancer.

**Figure 5:** ROC curve of the prognostic survival model for patients with TNBC with LM in the training cohort (a) and validation cohort (c). Survival curves of the high- and low-group were generated using the prognostic total score calculated from the nomogram in the training cohort (b) and validation cohort (d). ROC: receiver operating characteristic; LM: lung metastasis; TNBC: triple-negative breast cancer.

**Figure 6:** Calibration curves of the prognostic nomogram model for patients with TNBC with LM in the training cohort (a) and validation cohort (c) at 6, 12, and 18 months; the DCA curve of the prognostic nomogram model for patients with TNBC with LM in the training cohort (b) and validation cohort (d) at 6, 12, and 18 months. ROC: receiver operating characteristic; DCA: decision curve analysis; LM: lung metastasis; TNBC: triple-negative breast cancer.

**Figure 7:** ROC curves of independent risk factors for the prognosis of patients with TNBC with LM in the training cohort at 6 months (a), 12 months (b), and 18 months (c). ROC curves of independent risk factors for the prognosis of patients with TNBC with LM in the validation cohort at 6 months (a), 12 months (b), and 18 months (c). ROC: receiver operating characteristic; LM: lung metastasis; TNBC: triple-negative breast cancer.

**Table 1:** Clinical and pathological features of patients with TNBC.

	Training cohort (18936)	Validation cohort (8112)		*P* value
Age, years			4.953	0.084
≤40	2004 (10.6%)	933 (11.5%)		
41-60	9033 (47.7%)	3833 (47.3%)		
>60	7899 (41.7%)	3346 (41.2%)		
Tumour size, cm			0.033	0.983
≤5	16573 (87.5%)	7099 (87.5%)		
5.1-10	2005 (10.6%)	862 (10.6%)		
>10	358 (1.9%)	151 (1.9%)		
Race			0.293	0.864
White	13570 (71.7%)	5832 (71.9%)		
Black	3913 (20.7%)	1653 (20.4%)		
Other	1453 (7.7%)	627 (7.7%)		
Grade			8.162	0.043
I	358 (1.9%)	179 (2.2%)		
II	3249 (17.2%)	1321 (16.3%)		
III	15166 (80.1%)	6557 (80.8%)		
IV	163 (0.9%)	55 (0.7%)		
Histological type			<0.001	0.999
8500	16268 (85.9%)	6969 (85.9%)		
Other	2668 (14.1%)	1143 (14.1%)		
T stage			0.610	0.894
T1	7976 (42.1%)	3394 (41.8%)		
T2	8133 (42.9%)	3485 (43.0%)		
T3	1735 (9.2%)	747 (9.2%)		
T4	1092 (5.8%)	486 (6.0%)		
N stage			0.132	0.716
N0	12153 (64.2%)	5225 (64.4%)		
Nx	6783 (35.8%)	2887 (35.6%)		
Lung metastasis			1.635	0.201
No	18590 (98.2%)	7945 (97.9%)		
Yes	346 (1.8%)	167 (2.1%)		
Insurance			0.513	0.474
No	435 (2.3%)	198 (2.4%)		
Yes	18501 (97.7%)	7914 (97.6%)		
Marital status			0.274	0.601
No	8289 (43.8%)	3523 (43.4%)		
Yes	10647 (56.2%)	4589 (56.6%)		

**Table 2:** Univariate and multivariate logistic analyses of lung metastasis in patients with TNBC.

	Univariate analysis		Multivariate analysis	
	OR (95% CI)	*P* value	OR (95% CI)	*P* value
Age, years				
≤40				
41-60	1.061 (0.699-1.611)	0.782	1.295 (0.846-1.983)	0.233
>60	1.805 (1.202-2.709)	0.004	2.372 (1.561-3.602)	<0.001
Tumour size, cm				
≤5				
5.1-10	6.460 (5.091-8.195)	<0.001	1.220 (0.804-1.852)	0.349
>10	18.717 (13.567-25.821)	<0.001	2.411 (1.548-3.756)	<0.001
Race				
White				
Black	1.109 (0.722-1.704)	0.637		
Other	0.959 (0.737-1.249)	0.757		
Grade				
I				
II	1.411 (0.507-3.928)	0.509		
III	1.713 (0.635-4.621)	0.288		
IV	1.659 (0.367-7.501)	0.511		
Histological type				
8500				
Other	1.366 (1.036-1.801)	0.027		
T stage				
T1				
T2	3.806 (2.470-5.867)	<0.001	3.318 (2.138-5.149)	<0.001
T3	15.752 (10.120-24.518)	<0.001	9.164 (5.005-16.780)	<0.001
T4	43.134 (28.197-65.983)	<0.001	18.977 (11.179-32.217)	<0.001
N stage				
N0				
Nx	5.178 (4.068-6.590)	<0.001	2.182 (1.671-2.848)	<0.001
Lung metastasis				
No				
Yes	0.235 (0.073-0.760)	0.016		
Insurance				
No				
Yes	0.418 (0.258-0.679)	<0.001		
Marital status				
No				
Yes	0.562 (0.453-0.697)	<0.001		

**Table 3:** Clinical and pathological features of patients with TNBC with lung metastasis.

	Training cohort (336)	Validation cohort (144)
Age, years		
≤40	25	19
41-60	118	59
>60	193	66
Tumour size, cm		
≤5	149	69
5.1-10	126	49
>10	61	26
Race		
White	230	94
Black	84	36
Other	22	14
Grade		
I	2	3
II	38	19
III	291	118
IV	5	4
Histological type		
8500	271	120
Other	65	24
T stage		
T1	18	10
T2	91	39
T3	79	35
T4	148	60
N stage		
N0	71	36
N1	164	70
N2	28	15
N3	73	23
Surgery		
No	190	76
Yes	146	68
Radiotherapy		
No	4	2
Yes	332	142
Chemotherapy		
No	91	30
Yes	245	114
Bone metastasis		
No	242	89
Yes	94	55
Brain metastasis		
No	291	126
Yes	45	18
Liver metastasis		
No	240	110
Yes	96	34
Insurance		
No	17	9
Yes	319	135
Marital status		
No	198	84
Yes	138	60

**Table 4:** Univariate and multivariate Cox analyses of lung metastasis in patients with TNBC.

	Univariate analysis		Multivariate analysis	
	HR (95% CI)	*P* value	HR (95% CI)	*P* value
Age, years				
≤40				
41-60	1.382 (0.864-2.211)	0.177		
>60	1.532 (0.972-2.414)	0.066		
Tumour size, cm				
≤5				
5.1-10	1.191 (0.922-1.539)	0.180		
>10	1.061 (0.768-1.466)	0.719		
Race				
White				
Black	0.888 (0.529-1.491)	0.654		
Other	0.907 (0.690-1.191)	0.481		
Grade				
I				
II	1.146 (0.275-4.771)	0.851		
III	0.673 (0.167-2.711)	0.578		
IV	0.943 (0.172-5.158)	0.946		
Histological type				
8500				
Other	1.407 (1.054-1.878)	0.021	1.424 (1.061-1.910)	0.019
T stage				
T1				
T2	1.359 (0.783-2.361)	0.276		
T3	1.412 (0.808-2.470)	0.226		
T4	1.335 (0.781-2.284)	0.291		
N stage				
N0				
Nx	1.153 (0.864-1.539)	0.333		
Surgery				
No				
Yes	0.553 (0.436-0.701)	<0.001	0.619 (0.485-0.790)	<0.001
Radiotherapy				
No				
Yes	0.830 (0.309-2.231)	0.712		
Chemotherapy				
No				
Yes	0.399 (0.308-0.517)	<0.001	0.360 (0.273-0.474)	<0.001
Bone metastasis				
No				
Yes	1.487 (1.152-1.919)	0.002	1.386 (1.060-1.812)	0.017
Brain metastasis				
No				
Yes	1.970 (1.414-2.747)	<0.001	1.810 (1.281-2.558)	<0.001
Liver metastasis				
No				
Yes	1.833 (1.424-2.358)	<0.001	2.050 (1.576-2.667)	<0.001
Insurance				
No				
Yes	0.739 (0.452-1.209)	0.228		
Marital status				
No				
Yes	0.676 (0.532-0.857)	0.001	0.665 (0.522-0.849)	0.001

## Data Availability

The dataset from SEER database generated and/or analyzed during the current study are available in the SEER dataset repository (https://seer.cancer.gov/).
